# Development and Validation of Embedded Device for Electrocardiogram Arrhythmia Empowered with Transfer Learning

**DOI:** 10.1155/2022/5054641

**Published:** 2022-10-07

**Authors:** Rizwana Naz Asif, Sagheer Abbas, Muhammad Adnan Khan, Atta-ur-Rahman, Kiran Sultan, Maqsood Mahmud, Amir Mosavi

**Affiliations:** ^1^School of Computer Science, National College of Business Administration and Economics, Lahore 54000, Pakistan; ^2^Department of Software, Gachon University, Seongnam 13120, Republic of Korea; ^3^Department of Computer Science, College of Computer Science and Information Technology (CCSIT), Imam Abdulrahman Bin Faisal University (IAU), P.O Box 1982, Dammam 31441, Saudi Arabia; ^4^Department of CIT, The Applied College, King Abdulaziz University, Jeddah, Saudi Arabia; ^5^Department of Management, College of Business Administration, University of Bahrain, Zallaq, Bahrain; ^6^Slovak University of Technology in Bratislava, Bratislava 81107, Slovakia; ^7^Obuda University, Budapest 1034, Hungary; ^8^TU-Dresden, Dresden 01062, Germany

## Abstract

With the emergence of the Internet of Things (IoT), investigation of different diseases in healthcare improved, and cloud computing helped to centralize the data and to access patient records throughout the world. In this way, the electrocardiogram (ECG) is used to diagnose heart diseases or abnormalities. The machine learning techniques have been used previously but are feature-based and not as accurate as transfer learning; the proposed development and validation of embedded device prove ECG arrhythmia by using the transfer learning (DVEEA-TL) model. This model is the combination of hardware, software, and two datasets that are augmented and fused and further finds the accuracy results in high proportion as compared to the previous work and research. In the proposed model, a new dataset is made by the combination of the Kaggle dataset and the other, which is made by taking the real-time healthy and unhealthy datasets, and later, the AlexNet transfer learning approach is applied to get a more accurate reading in terms of ECG signals. In this proposed research, the DVEEA-TL model diagnoses the heart abnormality in respect of accuracy during the training and validation stages as 99.9% and 99.8%, respectively, which is the best and more reliable approach as compared to the previous research in this field.

## 1. Introduction

Electrocardiogram (ECG) is one of the best techniques to record the electrical signal to examine all the heart activities. If the heart is not working properly and activities are abnormal, then it would lead to serious and dangerous outcomes. Based on the World Health Organization (WHO) report, 30–40% of deaths in the entire world are due to cardiovascular diseases which is an alarming situation, and the ratio is increasing with the passage of time. This irregular functioning and abnormalities can be found by cardiologists [1]. Literature indicates that it is difficult to identify the accurate position and transition of ECG signals with one or a simple algorithm. Artificial intelligence (AI) is playing a vital role in the recognition of heart disease by using ECG readings. The ECG value depends on the techniques, algorithms, and different devices, which are used for detecting the signals of the ECG [2]. The rate of the heartbeat can be calculated by the QRS complex *R* peak, which represents the ECG signal per minute and shows the ventricular depolarization. The ECG wave along with its related trough and crest values such as QRS, QT, PR, and ST can explain the entire position of heart functionality [3]. The cardiologist can generate an ECG report in 3 seconds where the P wave can show atrial polarization having a duration of less than 0.12 s and amplitude of less than 2.5 mm. Then, the cardiac movement can take place from the atria to the ventricle in the PR interval of 0.12–0.2 s. The QRS complex represents the ventricular depolarization having a duration of 0.06–0.10 s. The healthy person has 0.10–0.12 s QRS, which is wider. After that, the *T* wave represents the ventricular repolarization, and it would have the same direction as the QRS. If the QRS complex is positive, the *T* wave will be positive, and if the QRS complex is negative, the *T* wave will be negative. The leading ST segment shows the interval between the depolarization and ventricular depolarization. The ST wave is a smooth wave line. So, the U wave shows the slower heart rate which is at the end leading from *T* [4]. It is important to go through the functioning of the heart and ECG before implementing it on any machine learning, deep learning, and transfer learning approach [3–5].

For the diagnosis of heart arrhythmia, the cardiologist can check the functionality of the heart and categorize it into different cardiovascular diseases upon symptoms, which can be helpful to cure the disease. The ECG analysis is one of the patterns which is applied to machine learning and deep learning to get a more precise result in a little span of time [3, 4, 6]. The study is a combination of hardware and software related to the deep learning approach. In the first part of the proposed model, build up hardware by using Raspberry Pi 3+, Arduino, a touch screen, and a heart monitor device to get the reading in real-time to create its dataset. The second part is to involve the software part, which involves different approaches of deep learning methods, and further use three databases, one from the Kaggle, i.e., Massachusetts Institute of Technology-Beth Israel Hospital (MIT-BIH Arrhythmia), the second one is own dataset named Real-Time Cardiac Arrhythmia (RT-CarArr), and the final dataset created by the combination of above two datasets, i.e., BIH-RT. The study has some parts to explain the proposed model for finding the accuracy in diagnosing ECG arrhythmia. The previous machine learning approaches to diagnose heart arrhythmia was found to be handcrafted and time-consuming. In the proposed model, the deep learning approach enhanced the accuracy and speed as compared to the machine learning methodology. In this regard, the transfer learning method AlexNet widens the research, proves the accuracy, and maximizes the results in diagnosing heart problems and abnormalities. The introduction is given in Section 1, and in Section 2, literature review, limitations, past work, and achievements are provided. Last but not the least, this will have to cover the proposed model's working performance, methodology, research tools and material, and conclusion.

## 2. Literature Review

The ECG signals which can provide the actual beat of the heart in the peak *R* in the time series have been analyzed with machine learning techniques [7]. An innovative deep learning approach and techniques help to detect abnormalities spontaneously. Deep learning made a progress in the AI field, and it could be effective for the image analysis of ECG [7, 8]. The multidimensional work (1D, 2D, and 3D) is possible with the convolutional neural network (CNN), where the 1D is limited to time series data, which are less effective as compared to 2D CNNs. So, the time series in 2D is good for machine learning algorithms [3, 9, 10]. Hence, the 2D images as the input can be applied to the ECG to make it a learning perspective and can be able to extract the features for the ECG representation. This one representation makes it possible to develop cardiovascular disease (CVD) through different automated systems. The cardiologist took some time to find the arrhythmia disease, could be an hour of observation for the analysis of ECG. The arrhythmia detection can be performed with the help of time-varying and morphological features by using hybrid feature classification. The various classification will control different kinds of wavelengths, which can occur in arrhythmia [5, 11, 12]. The IoT helped to make it possible to go through the hardware and software together with cloud computing. The ECG signal analysis worked with the classification and real-time implementation and linked with a variety of hardware (Arduino, Bluetooth, cloud servers, and phone with ECG monitor) to work parallel with the software as transfer learning and machine learning to get the accurate or required results [6, 13]. There is more work with ECG and blood pressure (BP) and their relationship; the BP value can be detected with numeric data and based on feature extraction with a machine learning model. This method was applied to estimate arterial pressure, systolic BP (SBP), and diastolic BP (DBP) by using the ECG sensor [2, 14, 15]. The classification of ECG can also be carried out with the pattern recognition method and artificial neural network (ANN) in various research studies. Moreover, the ANNs method enhanced the QRS peak detection by utilizing the multilayer perception [16, 17]. Here, the preceptor behaved like a classifier that helped to distinguish the wavelength of the normal and abnormal ECG signal reports in the form of an image to a cardiologist to read and suggest to the patient the current position either healthy or unhealthy, in the respect of heart functionality. Improvement has been seen in the ECG while using a mixture of expert (MOE) with ECG classification. In this machine learning technique, the real-time patient data can collaborate with the large dataset to get the MOE classifier. For more accuracy in the short span, the self-organizing map (SOM) is used to get the more accurate result for different kinds of heart diseases [15, 16].

Another study about the ECG has been seen in the biosignal as well; when a person has anxiety and pressure while driving a car, the supervised machine learning algorithm used the ECG movement and signals' information for biosignals and proved 72.5% accuracy [8, 16, 17]. The detection of Alzheimer's disease uses the synchronization measures acquired with magnetoencephalography. In this way, the novel deep learning model is proposed and based on different blocks of the pooling layers, 2D convolution, and batch normalization. This model is designed to avoid overfitting, as there are massive images (25755) with few samples (132 patients). To solve the issue is to outfit the submodels with the sharing weight, and the final stage can be achieved by performing the average of submodels. Therefore, each submodel can receive the random permutation of features, which correspond to the neural activity and are arranged in the matrix form as a 2D image, which is further sorted out by a 2D convolution network. Their proposed model is a binary classifier and compared to the machine learning and deep learning approach by obtaining the best classification result with an average F1 score of 0.92 [3, 18]. Singh proposed an attention-based convolutional model to diagnose atrial fibrillation from wearable ECG. The features are extracted by using the convolution layer and classifying the atrial fibrillation. The model was tested on four databases and achieved a classification performance of 99.25% for precision, 99.25% for accuracy, and 99.50% for recall, respectively [19]. Lopez-Martin et al. presented a novel contrastive learning design and the loss function. The novel classifier was suitable for unstable and noisy datasets for intrusion detection [20].

The two main things are involved in it: one is accuracy and performance metrics and the other is computational knowledge and complexity (big O notation). The other limitation is the design and assembling techniques to operate the method or algorithm. The improvements and updating should have been seen in the datasets of the ECG. The doctors and researchers, using the portable and wearable ECG, should have to share ideas to make it real-time reliable and more effective [2, 14, 15]. The transfer learning approach can give more precise and accurate data in terms of electric ECG signals and by using MIT-DB and ECG-ID, got the satisfactory result of 97.7% for MIT-DB and 94.4% for ECG-ID and provides the qualitative result to prove the uniqueness [12, 16, 21, 22]. Jignesh et al. proposed the transfer learning of inception V3 while using the face mask for the detection of the face and achieved remarkable accuracy in testing and training [23]. The transfer learning approach is also helpful in other fields of the biomedical such as in breast cancer. Gelan Ayana et al. proposed the ImageNet transfer learning method to detect breast cancer for detection and diagnosis and achieved accuracy better as compared to the previous research [24–27]. The deep learning approach with the recurrent neural network (RNN) is useful in the ECG rhythm classifier for the sequence modeling of imbalanced data and further compared the performance of the RNN with the long short-term memory (LSTM) and gated recurrent unit (GRU) and observed that the LSTM technique is the latent method for the sequential data with an accuracy of 97.7% [28–31]. In addition, researchers proposed the validation of ECG-derived sleep architecture and ventilation in sleep apnea and chronic fatigue syndrome and analyzed the result by using the kappa score, which is 0.68, 0.85, and 0.69 for different classes [30]. Guangyu Xu proposed that the IoT built an ECG monitoring framework to improve the accuracy of the system with entire devices [22, 32–34]. An updated, comprehensive architecture for the Internet of Things devices is built on modernized blockchain models. The authors of [35] devised an intelligent way to combine IoT and blockchain in autonomous integrated sewage management. The model and framework can examine and compare various current blockchain strategies. The term “remote patient monitoring” describes keeping track of a patient's health through various digital communication channels. It uses mobile devices to collect and report on various health parameters, including those connected to the Internet of Things or the patient's body. The blockchain has been beneficial for acquiring, sharing, and storing data. It has been suggested to use IOB Health, Ethereum smart contracts, and hyperledger fabric technology [36]. Electronic health records (EHRs), electronic medical records (EMRs), remote patient monitoring, the pharmaceutical supply chain, and health insurance claims are some of the critical healthcare applications for blockchain. There is a difference between an electronic health record (EHR) and an electronic medical record, even though they are frequently used interchangeably. An EMR is similar to a digital patient chart or prescription because it records a patient's medical history and cares at a single medical facility. An electronic health record more accurately depicts a patient's overall health than it is by a paper one. Applications for EMR and EHR have been created that use and support blockchain technology Med Rec, FHIR Chain, MedShare, Ethereum applications, Med Block, and Block HIE [37]. We created an SVM-merged AlexNet classifier to handle so many attributes quickly. SVMs accelerate the hyperplane convergence in the fully connected layers of the AlexNet. Because we did not wish to begin from scratch, we used transfer learning to partially freeze the initial layers and fine-tune the features that were learned [38]. We used our architectural framework to evaluate it against the best work produced up to that point. The proposed architecture was classified more accurately than the top-ranked architectures, and its implementation took much less time. Due to this, it is a great choice when time is of the essence. The proposed algorithm [4] could be used to create better AI solutions for maternal and infant care.

In [39], the authors proposed and discussed how our design addressed typical security concerns and proposed a novel way to use blockchains to secure healthcare data. Numerous benefits exist for the proposed architecture, including increased security against known threats, decreased traffic growth, increased transparency, instantaneous traceability, and robustness. Our architecture, according to testing, reduces network traffic by a factor of 10 and speeds ledger updates by 63%. In [40], a translational combination of deep learning algorithms and CTG data was proposed, and it showed promising results with respect to accuracy and processing time. They improved the necessary time-performance metrics in medical settings. The algorithm outperformed the best architectures currently on the market with a sensitivity of 96.67%. Performance comparison of 2D and 3D CNN architectures is done for early Alzheimer's disease symptom detection [41]. We divided people into the four groups of Alzheimer's disease (AD), non-Alzheimer's disease (NC), mild cognitive impairment (MCI), and AD using a five-fold CV method for selecting hyperparameters. Both “start from scratch” and “transfer learning” methods were used in the training of the participants. We improved the accuracy of the AD/NC classification task, the AD/MCI classification task, the NC/MCI classification task, and the AD/NC/MCI classification task using 3D CNN architectures, bringing them to 89.21%, 71.70%, 62.25%, and 59.73%, respectively. Our findings show the importance of starting from scratch in the higher domain by demonstrating that CNN architectures perform best in 3D space. The suggested forensic analysis system [42] covers IoT devices' constrained memory and resources. With the proposed forensic system, identifying the issue with Internet of Things devices in a wired environment is now simpler and faster than ever. Network traffic is sent to the logging server, where it is analyzed using previously defined rules without preventing devices from communicating. These malicious traffic logs are kept on file by the forensics server, which makes it possible for them to be recreated differently. A dataset is also produced when the Internet of Things-enabled devices record an attack. For attack detection, various machine learning models are trained and assessed. The decision tree algorithm performed admirably, with a 97.29% accuracy rate. Our plan is immediately tested when a Raspberry Pi camera is connected to the network. The decision tree's 96.01% accuracy reduced the power of machine learning models.

Some of the problems related to animal identification may be resolved with the help of the proposed research, artificial intelligence, and artificial general intelligence fields. Machine learning and federated learning are additional provider domains that could help with animal identification. The problem we just discussed might be simulated using real-time data in the future. To obtain the most accurate results, several AI-based techniques (RF, VGG-16, SVM, SMOTE, ECNN, CNN, NB, and XGBoost) were applied to various datasets. The accuracy percentages for RF, VGG, SVM, SMOTE, ECNNs, CNN, NB, and XGBoost are 98%, 97%, 92%, 90%, 88.8%, 82.15%, 81.5%, and 78.9%, respectively [43, 44]. In comparison, the machine learning and deep learning approach along with the ECG work, as well as compared to the ECG signals themselves. From the limitation perspective, machine learning needs higher computational knowledge, and the cost is high for the processors to operate [21].

### 2.1. Limitations of the Related Work

There are a few limitations regarding the previous research, as given in Table 1.

- The dataset is not fused and augmented
- The new real-time dataset is not generated
- The proposed model is more accurate compared to the previous one which is comparatively showing less accuracy
- In the previous research, there is not any hardware implementation and ECG signal data have not been taken in real-time

### 2.2. Our Contributions

The major contribution of the study is as follows:

- In the past research, the datasets are feature-based and handcrafted; in the proposed model, the deep learning approach (AlexNet) is applied instead of machine learning to get a more precise result.
- The real-time hardware and software are designed and implemented to get accurate results of heart arrhythmia

## 3. Proposed Model

According to the WHO, a lot of patients especially those under the age of 40 plus can have cardiovascular disease and arrest which be for a variety of reasons. The best knowledge of ML and DL with the help of different algorithms made it possible to work in more advanced ways along with the usage of innovative devices. Doctors could monitor the patients in real-time and can evaluate the sign of the diseases with the help of ECG reading with the peak values [17, 45, 46]. The research first initiates the understanding of the working of the heart and ECG electric signals and terminology to detect and diagnose cardiac arrhythmia. Three databases are used are MIT-BIT Arrhythmia with five classes (F, N, Q, S, and V), RT-CarArr with two classes (healthy and unhealthy), and BIH-RT having five classes with the combination of MIT-BIT Arrhythmia and RT-CarArr. The proposed DVEEA-TL model is comprised of two parts, namely, hardware and software. The focus is to diagnose cardiac arrhythmia by using a transfer learning model, and with the help of hardware, it is possible to get real-time images and do the IoT. Initially, the actual and main MIT-BIH Arrhythmia dataset has been taken from Kaggle, and then, the real-time dataset for the healthy and unhealthy person has been generated with the help of the proposed embedded hardware (Arduino, heart rate monitor chip, 7″ touch screen with Raspberry Pi, wires, electrode pads, and so on) and able to take the reading from this 7″ touch screen and later check against the proposed system if the person is healthy or unhealthy. Furthermore, the MIT-BIH dataset and the own created dataset of healthy and unhealthy patients must augment in python with the help of Keras. Then, we fused both datasets. Later, the fused dataset BIH-RT can get trained, validate, and apply performance in terms of accuracy.

### 3.1. Hardware Implementation of the Proposed DVEEA-TL Model

The emulation board and software (Arduino IDE) are compatible, in respect of hardware initiatives, and connect with the ECG sensor (AD8232) with compatible clips, cup electrodes, and ECG cables [1, 7].  Figure 1 shows the hardware connectivity for the proposed DVEEA-TL model. Furthermore, to display the ECG signal reading from the emulator, there is ultimate need for the monitor, and for that purpose, the Raspberry Pi 3.0+ with the 7″ monitor touch screen is used which is portable and easy to operate [1, 2]. The real-time dataset RT-CarArr has been created by using the hardware, and it is comprised of 2 classes, namely, healthy and unhealthy. Whenever the whole hardware is set up, apply the three electrodes in three different places of the patient, commonly at the left arm, right arm, and left leg, as shown in Figure 1. The ECG signals will be taken from the body through electrodes and passed to AD8232, and through Arduino programming, the signals are taken and displayed on the 7″ screen of Raspberry Pi 3B+. If the patient does not have any heart problem, then it will show the frequency 360 Hz and bandwidth range from 0.5 to 40 Hz in 600 s. Finally, at this stage, the analog signals are obtained. Furthermore, the signals are compacted and reduced by fast Fourier transform (FFT) and get more refined without noise signals [1].

### 3.2. Software Implementation of the Proposed DVEEA-TL Model

The computer-based software such as python and MATLAB 2021a helped to work with the algorithm, and different deep learning approaches MATLAB and made it possible to get the prerecorded ECG data from the available database from Kaggle and own created databases which can be preprocessed according to the required dimensions for these methods.  Figure 2 shows the entire architecture of the DVEEA-TL model from hardware to software implementation with transfer learning methodology.

#### 3.2.1. Dataset

As discussed earlier, all three datasets are used; one dataset is from Kaggle [47], the other is own created, and the third one is the combination of the first two datasets. The augmentation and fusion of data have been carried out against the newly generated dataset. Then, preprocess the dataset and convert it into the ECG classification by using the deep learning method AlexNet. For this purpose, the required dataset has been taken from the BIH-RT database with N (normal beat), S (supraventricular ectopic beat), V (ventricular ectopic beat), F (fusion eat), and Q (unknown beat) [47]. The number of MIT-BIH Arrhythmia for signals has been recorded for each category in this dataset as N (1500), S (3879), V (3647), F (2500), and Q (3500), respectively, which is further augmented and produce more images according to the requirement, and for the further testing, Table 2 presents the new number of samples for this MIT-BIH Arrhythmia database. In Table 3, two classes are introduced as healthy and unhealthy in the real-time database RT-CarArr with 1500 each number of images. Then, after the data fusion of both datasets, Table 4 shows the new database BIH-RT, which is generated with overall 18026 images. Furthermore, the real-time ECG images are taken with the help of hardware and extracted through frames and compressed the signals through FFT, and then, preprocess the images. Tables 2–4 show the actual picture of all datasets which are used in the proposed DVEEA-TL model along with several classes and a number of ECG images. In the proposed DVEEA-TL model, overall, 18026 images with 5 classes are used for preprocessing, training, and validation. The whole structure of hardware and software is the best combination of innovative real-time ECG arrhythmia analysis, diagnosis, and implementation [5, 17].

#### 3.2.2. Transfer Learning Architecture

The software implementation is the essential and basic requirement of ECG arrhythmia where the transfer learning method helped to find the required accuracy in diagnosing the ECG performance and find the abnormalities if found by the proposed method.  Figure 3 shows the entire system in the simplest way to show the flow of working as “input data and collection,” “preprocessing,” “training,” “validation,” “performance,” and “implementation” of the proposed DVEEA-TL model.

The pseudocode of the proposed DVEEA-TL model is given in Table 5.

The deep learning approach is a widely used technique in a variety of fields such as health, transportation, agriculture, gaming, aeronautics, and so on [17]. Different pretrained transfer learning methods and models are used in this respect. Here, in the proposed DVEEA-TL model, by using AlexNet, cardiac arrhythmia can be classified and diagnosed. AlexNet is the pretrained model and has 25 layers. The images were resized according to the AlexNet parameters or dimensions as 227 × 227 × 3. The preprocessing of fused data of 5 different classes shown in Figure 4 has been taken from the database BIH-RT.

After preprocessing, the fine-tuning method was applied to images, and according to the requirement, layers have been changed. Then, trained and validated all the images with a 70 : 30 ratio. The proposed DVEEA-TL model showed 99.9% with training and 99.8% with validation, respectively.  Table 6 provides the number of images used for training and validation purposes.

Based on the prerequisite and the properties of the proposed DVEEA-TL model, the last three layers are changed, as shown in Figure 5. Figure 5 shows the used architecture in the proposed DVEEA-TL model.  Figure 6 shows the accuracy and loss rate of the proposed DVEEA-TL model.

## 4. Simulation and Results

A matrix comprises accuracy, classification miss rate, sensitivity, precision, false positive ratio, false negative ratio, F1 score, Mathew correlation coefficient (MCC) analysis, specificity, and kappa score are used to evaluate the overall performance of the fine-tuning approach. The assessment and development of the entire program are to be carried out in the MATLAB 2021a with 11th Gen Intel(R) Core (TM) i5-1135G7 @ 2.40 GHz computer processor, 8.00 GB RAM, and 1 TB hard disk along with also tested on Raspberry Pi 3.0+, Arduino, and heart monitor on run time. Performance evaluation of algorithms is evaluated with different statistical parameters as shown in the following equations adapted from [27–33, 45]:

(1) $$\begin{array}{c} Accuracy=\frac{O_{ri}+O_{rk}/I_{ri}+I_{ik}}{O_{ri}/I_{ri}+\sum_{j=1}^{n}\left(O_{ri},j\neq i\right)/I_{rj}+O_{rk}/I_{rk}+\sum_{l=1}^{n}\left(O_{rl},l\neq k\right)/I_{rk}}where\;l,j,i,k=1,2,\ldots ,m\text{,} \end{array}$$

(2) $$\begin{array}{c} Miss\;rate=\frac{\overset{n}{\underset{l=1}{\sum }}O_{rl\;,l\neq k}/I_{rk}}{\;\sum_{l=1}^{n}\left(O_{rl\;,l\neq k}\right)/I_{rk}+O_{ri}/I_{ri}}where\;l,j,i,k=1,2,\ldots ,m\text{,} \end{array}$$

(3) $$\begin{array}{c} True\;positive\;rate/recall=\frac{\;O_{ri}/I_{ri}}{\;O_{ri}/I_{ri}+\sum_{l=1}^{n}\left(O_{rl},l\neq k\right)/I_{rk}}where\;l,j,i,k=1,2,\ldots ,m\text{,} \end{array}$$

(4) $$\begin{array}{c} \frac{True\;negative\;rate}{Sensitivity}=\frac{O_{rk}/I_{rk}}{O_{rk}/I_{rk}+\sum_{j=1}^{n}\left(O_{rj},j\neq 1\right)/I_{rj}}where\;k,j=1,2,\ldots \ldots ,m\text{,} \end{array}$$

(5) $$\begin{array}{c} Precision=\frac{\;O_{ri}/I_{ri}}{\;O_{ri}/I_{ri}+\sum_{j=1}^{n}\left(O_{rj},j\neq 1\right)/I_{rj}}where\;j,i=1,2,\ldots ,m\text{,} \end{array}$$

(6) $$\begin{array}{c} False\;omission\;rate=\frac{\overset{n}{\underset{l=1}{\sum }}\;O_{rl\;,l\neq k}/\;I_{rk}}{\sum_{l=1}^{n}\left(O_{rl\;,l\neq k}\right)/I_{rk}+O_{rk}/I_{rk}}where\;l,k=1,2,\ldots \ldots ,m\text{,} \end{array}$$

(7) $$\begin{array}{c} False\;discovery\;rate=\frac{\overset{n}{\underset{j=1}{\sum }}\;O_{rj\;,j\neq i}/I_{rj}}{\;O_{ri}/I_{ri}+\sum_{j=1}^{n}\left(O_{rj},j\neq i\right)/I_{rk}j}where\;i,j=1,2,\ldots \ldots ,m\text{,} \end{array}$$

(8) $$\begin{array}{c} F\;0.5\;score=1.25\;x\;precision\;x\frac{recall}{0.25\;x\;precision+recall}\text{,} \end{array}$$

(9) $$\begin{array}{c} F1\;score=2\;x\;precision\;x\frac{recall}{precision+recall}\text{,} \end{array}$$

(10) $$\begin{array}{c} MCC=\frac{\left(TP\;x\;TN\right)-\left(FP\;x\;FN\right)}{\sqrt{\left(TP+FP\right)\left(TP+FN\right)\left(TN+FP\right)\left(TN+FN\right)}}\text{,} \end{array}$$

(11) $$\begin{array}{c} Kappa\;score=\frac{p_{o}-p_{e}}{1-p_{e}}\text{,}=1-\frac{1-p_{o}}{1-p_{e}}\text{.} \end{array}$$

MCC is used to measure the microaveraging for each class and then calculate the statistics. The MCC values used the true positive (TP), true negative (TN), false positive (FP), and false negative (FN) for each class, and the final statistic value is given in Table 7. With the help of the kappa score, the classification performance can be measured by using the metrics, and it can show the observed and estimated value and the probability of its existence. Kappa score is always equal to “1” or less than “1.” The values against kappa analysis are given in Table 8. The performance of five different classes is observed by using the accuracy, sensitivity, classification miss rate, and specificity. The confusion matrix in Figures 7 and 8 shows the class-level comparison applied to transfer learning which is used in architecture. All the classes showed different values as the training set values for F are 899 TP, 4 FN, 1 FP, and 4554 TN with an overall accuracy is 99.91%, as shown in Figure 7. The matrix value for N is 1164 TP, 3 FN, 0 FP, and 4290 TN with an overall accuracy is 99.94%.

Hereafter, the confusion matrix value for Q is 1094 TP, 0 FN, 6 FP, and 4358 TN with an overall accuracy is 99.89%. So, the matrix value for S is 1200 TP, 0 FN, 0 FP, and 4258 TN with an overall accuracy of 100%. Last, the matrix value for Q is 1094 TP, 0 FN, 0 false positive, and 4364 true negative as shown in Figure 8. The simulation result of all classes of transfer learning is given in Tables 7 and 8, and it represents the accuracy, classification miss rate, sensitivity, specificity, precision, false negative ratio (FNR), and false positive ratio (FPR) of all five ECG classes.

## 5. Comparative Analysis of the Proposed Model

Table 9 provides the comparison result of the proposed DVEEA-TL model with the literature. This proposed model is a combination of hardware and software, which made it distinct from the previous research. Furthermore, the real-time own dataset, data fusion, and data augmentation are the achievements of this study as well. In the comparative analysis, it observed that the proposed DVEEA-TL model is giving the reckless and most trustworthy result as compared to previously published approaches.

## 6. Conclusions

In the proposed model, ECG devices, the algorithm, dataset, and ecological and financial factors all play an important role in determining the efficiency of ECG analysis. The more critical thing in heart arrhythmia is to diagnose in the early stages to save the life, and the ECG is the best step or ointment to check the functioning of the heart ECG signals. In the proposed DVEEA model, five different classes have been classified, preprocessed, trained, and validated in the knowledge of the artificial network. Furthermore, the augmented and fusion of data improved the probability of accuracy. The proposed model DVEEA-TL has the combination of hardware along with the software in MATLAB 2021a, Python, and Arduino working, and the datasets are trained on 10 epochs. Working on different layers helped to diagnose the ECG arrhythmia that gives a 99.9% and 99.8% training accuracy and validation accuracy, respectively, which is an excellent and outstanding result for the life-threatening cardiac disease. The proposed DVEEA-TL model showed remarkable accuracy, but there are still some variations and limitations, which must be in consideration and work in the future. For this model, the computation processing is high and consumes time to train the datasets of the ECG images. Furthermore, in the future, we can improve the computation processing to use the AWS or GPU, instead of the CPU to get the training at an enormous speed. An innovative and secure federated deep learning approach can be applied further to the proposed model to make it more consistent and steady in the medical sciences.

## Figures and Tables

**Figure 1:** Hardware connectivity of the proposed DVEEA-TL model.

**Figure 2:** The proposed DVEEA-TL architecture.

**Figure 3:** Proposed DVEEA-TL model.

**Figure 4:** Samples of 5 classes after preprocessing.

**Figure 5:** Transfer learning architecture of the proposed DVEEA-TL.

**Figure 6:** Accuracy and loss rate of the proposed DVEEA-TL model.

**Figure 7:** Confusion matrix (training of ECG dataset).

**Figure 8:** Confusion matrix (validation of ECG dataset).

**Table 1:** Limitations of the related work and its outcomes.

Studies	Dataset	Technique	Outcomes	Limits
Yeh et al. [1]	Private and PTB DB	ResNet, AlexNet, and SqueezeNet	Accuracy and kappa statistics of ResNet, AlexNet, and SqueezeNet in ECG waveform classification (0.97, 0.96), (0.96, 0.95), and (0.75, 0.67).	(i) No data augmentation, (ii) less accurate, and (iii) worked on waveform classification

Wasimuddin et al. [2]	ECG-ID	CAD and machine learning approach	CAD and machine learning approach working on 2D image based on classification and worked on the *R* peak of the ECG and showed an accuracy of 98.5%.	(i) Handcrafted features, (ii) small dataset, and (iii) accuracy is remarkable but slow because of handcrafted features

Hsu et al. [7]	MIT-BIH	AlexNet and ResNet 18	ECG into the fingerprint by using the transfer learning methods and proved the predicted accuracy of 94.4%.	(i) No data augmentation and (ii) handcrafted features

Elgendi and Menon [8]	Private	Machine learning approach	Supervised ML algorithms confirmed that ECG is an optimal wearable biosignal for assessing driving stress, with an overall accuracy of 75.02%.	(i) Low accuracy, (ii) augmentation not performed, and (iii) handcrafted features

Gaddam and Sreehari [12]	MIT-BIH	AlexNet	Transferred deep learning convolution neural net with 1D and 2D structure with 95.6% accuracy.	(i) Augmentation not performed and (ii) low accuracy

Simjanoska et al. [14]	4 private datasets used	Machine learning	The proposed method achieved 8.64 mmHg of the mean absolute error in the case of SBP.	(i) Handcrafted and (ii) low accuracy

Acharya et al. [15]	PTB DB	CNN layers	CNN for automated detection of myocardial interaction using ECG signals, and inferred the data with noise (93.5%) and without noise (95.22%).	(i) Low accuracy and (ii) less number of classes

Tomer Golany [21]	Private	GAN-based generative models such as GAN, DCNN, SIMCGAN, and SIMDCGAN.	Simulator-based network for ECG to improve deep ECG classification was used and compared all GAN-based models to find the accurate result of ECG and got SIMDCGAN as a refined and result-oriented model.	(i) Low accuracy, (ii) augmentation not performed, and (iii) handcrafted features

Sehirli et al. [28]	PTB-XL	RNN (LSTM and GRU)	Compared the performance of the RNN with the long short-term memory (LSTM) and gated recurrent unit (GRU) and then observed that the LSTM technique is the latent method for the sequential data and time series with the accuracy of 97.7%.	(i) Less accurate, (ii) small dataset, and (iii) augmentation not performed

Strodthoff et al. [33]	PTB-XL	ResNet and inception	Deep learning of ECG analysis by using datasets showed an 89.8% result.	(i) No augmentation and (ii) low accuracy

Rahman et al. [45]	MIT-BIH	CAA-TL model (deep learning)	Different transfer learning approaches analyzed with data augmentation achieved 98.38% accuracy.	(i) No data fusion, (ii) low accuracy, and (iii) no hardware implementation

**Table 2:** MIT-BIH Arrhythmia augmented dataset (Kaggle) [47].

No.	Feature name	No. of samples
1	N (normal beat)	1500
2	S (supraventricular ectopic beat)	3879
3	V (ventricular ectopic beat)	3647
4	F (fusion beat)	2500
5	Q (unknown beat)	3500
	Total number of images	15026

**Table 3:** RT-CarArr augmented dataset.

No.	Feature name	No. of samples
1	Healthy (normal beat)	1500
2	Unhealthy (fusion beat)	1500
	Total number of images	3000

**Table 4:** Augmented and fused datasets BIH-RT (real-time).

No.	Feature name	No. of samples
1	N (normal beat)	3000
2	S (supraventricular ectopic beat)	3879
3	V (ventricular ectopic beat)	3647
4	F (fusion beat)	4000
5	Q (unknown beat)	3500
	Total number of images	18026

**Table 5:** Pseudocode of the proposed DVEEA-TL model.

S no.	Step
1	Begin
2	Input ECG data
3	Augmentation and data fusion
4	Preprocess ECG data
5	Load data
6	Load pretrained model
7	Modified the model
8	Trained the modified model
9	Validate the modified model
10	Perform performance evaluation
11	End

**Table 6:** The proposed DVEAA-TL model used data division during training and validation.

Classes	Total no. of instances (100%)	Training instances (70%)	Validation instances (30%)
Q	3647	2552	1095
N	3879	2715	1164
F	3000	2100	900
V	3500	2450	1050
S	4000	2800	1200
Total	18026	12617	5409

**Table 7:** Class-wise training and validation results of the proposed DVEEA-TL model.

T	Evaluation matrix	F	N	V	Q	S
		Fusion beat (%)	Normal beat (%)	Ventricular beat (%)	Unknown beat (%)	Supraventricular beat (%)
Accuracy	Training	99.91	99.95	99.88	100	100
	Validation	99.81	99.78	99.82	100	100

Classification miss rate	Training	0.09	0.05	0.12	0	0
	Validation	0.19	0.22	0.18	0	0

Sensitivity	Training	99.56	99.74	100	100	100
	Validation	98.90	100	100	100	100

Specificity	Training	19.74	27.13	25.07	25.07	28.19
	Validation	20.03	34.93	23.69	25.37	28.55

Precision	Training	99.89	100	54.70	100	100
	Validation	100	100	99.04	100	100

FPR	Training	0.80	0.73	0.75	0.75	0.72
	Validation	0.80	0.65	0.76	0.75	0.71

FNR	Training	0.004	0.002	0	0	0.004
	Validation	0.01	0	0	0	0

**Table 8:** Proposed DVEEA-TL model' overall results.

Performance matrices	Training (%)	Validation (%)
Accuracy	99.9	99.8
Classification miss rate	0.05	0.07
Sensitivity	99.8	99.7
Specificity	21.09	26.5
Precision	90.9	99.80
F1 score	0.98	0.97
FPR	0.75	0.73
FNR	0.002	0.002
MCC	99.2	98.5
Kappa score	0.98	0.97

**Table 9:** Proposed DVEEA-TL model compared with the state-of-the-art literature.

Studies	Hardware implementation	Data augmentation	Data fusion	Datasets	Method	Findings
Yeh et al. [1]	Yes	No	No	PTB DB	ResNet, AlexNet, and SqueezeNet	Predicted accuracies: 97%, 95%, and 75%
Wasimuddin et al. [2]	No	No	No	ECG-ID	CAD and machine learning	Predicted accuracy: 98.5%
Vijayakumar et al. [6]	No	No	No	No	Feature extraction to remove noise	Predicted accuracy: 96.5%
Hsu et al. [7]	No	No	No	MIT-DB	AlexNet and ResNet	Predicted accuracy: 94.4%
Gaddam and Sreehari [12]	No	No	No	MIT-DB	AlexNet	Predicted accuracy: 95.6%
Simjanoska et al. [14]	No	No	No	PTB DB	ML-train-validation-test evaluation	Predicted accuracy: 98%
Acharya et al. [15]	No	No	No	PTB DB	CNN layers	Predicted accuracy: 93.5% (for noise data) Predicted accuracy: 95.22% (for non-noise data)
Hammad et al. [17]	No	No	No	PTB	ResNet model	Predicted accuracy: 98.85%
Golany et al. [21]	No	No	No	MIT-DB	GAN-based model	Predicted accuracy: 97.5%
Sehirli et al. [28]	No	No	No	PTB-XL	RNN (LSTM and GRU)	Predicted accuracy: 97.7%
Strodthoff et al. [33]	No	No	No	PTB-XL	ResNet and inception	Predicted accuracy: 89.8%
Rahman et al. [45]	No	Yes	No	MIT-BIH	CAA-TL model (deep learning)	Predicted accuracy: 98.38%
Proposed DVEEA-TL model	Yes	Yes	Yes	BIH-RT (real-time dataset)	Transfer learning (AlexNet)	Training (99.9%)
						Validation (99.8%)

## Data Availability

The data used to support the findings of this study are available from the corresponding author upon request.
